The article "Is Equity Crowdfunding the Leapfrog to Companies' Success? Financial Performance in China" was published in 2022. Journal: Comput Intell Neurosci.

# Is Equity Crowdfunding the Leapfrog to Companies' Success? Financial Performance in China

**DOI:** 10.1155/2022/7814550

**Published:** 2022-08-29

**Authors:** Chang Jiang, Raquel Pérez-Estébanez, Elena Urquía-Grande

**Affiliations:** Faculty of Economics & Business, Department of Financial Administration and Accounting, Complutense University of Madrid, 28223 Madrid, Spain

## Abstract

As the fastest-growing crowdfunding model, equity crowdfunding (ECF) brings high returns and uncertainty. In this context, it is crucial to understand these crowdfunding projects' actual performance. Since ECF is currently in the early stage of integration, there are still a lot of risk issues, such as the uncertainty of equity structure, capital supervision, or project management. Therefore, this paper develops a new profitability indicator, “return on registered capital,” to test its impact on the ECF project's actual return. This paper studies which factors affect the financial performance of ECF projects through the traditional statistical model and a deep neural network (DNN) model. There is evidence that return on registered capital affects the actual return of the project. At the same time, the company's operating time and the number of employees had an unexpected effect on project performance. In addition, the recognition accuracy of the DNN model in this study exceeds 97%, which affirms the applicability of the DNN model in the analysis of ECF success factors. This paper also uses tenfold cross-validation to prove that deep learning has certain advantages in this topic's accuracy and generalization error. This study explores whether company representatives' gender and knowledge level affect project performance. The results will be described in detail in the paper.

## 1. Introduction

The Internet has changed the way of social communication and people's way of life, and it also had a massive impact on the financial industry's innovation. Entrepreneurs, especially in SMEs, have difficulty obtaining business loans or investments in the early stages of their business, resulting in many projects ultimately failing. With the continuous development of Internet finance, many new financing methods have emerged. Crowdfunding is one of them, it is a “preconsumption” model that applies to ordinary backers by raising their investments to fund projects, and they can also earn future profits through projects [1].

Generally, scholars divide crowdfunding into four categories: donation-based, reward-based, equity, and lending. Equity crowdfunding (ECF) has developed rapidly in recent years as a subcategory of crowdfunding. Vulkan et al. [2] pointed out in their research that the development of ECF will pose a massive challenge to venture capital and business angel financiers in the future. Several years have passed, and until now, facts have proved that ECF has substantially impacted traditional investment fields.

The article "Is Equity Crowdfunding the Leapfrog to Companies' Success? Financial Performance in China" was published in 2022. Journal: Comput Intell Neurosci.

The existing research on the ECF theme has developed rapidly in recent years. On the one hand, some researchers have studied ECF development, such as ECF and pervasive finance [3], market size and geographical distribution [4], and plagiarizing product ideas [5].

On the other hand, some researchers have paid attention to ECF's performance and success factors' internal activities. This direction has become a hot spot for ECF research nowadays. Some researchers focus on the project sponsors' social capital [6], the static factors like the ultimate campaign outcome of innovative companies [7, 8], and the return on investment [9, 10] all the factors on project success.

As a new investment and financing mechanism, entrepreneurs who need funds can use ECF for rapid financing. The public can also use ECF to support projects that require funds and obtain high returns. Also, it brings great uncertainty. Therefore, the present research proposes a new idea to improve the performance research of ECF. Unlike most existing studies, it has not focused on ECF projects' performance in the raising or financing process. This paper concentrates on the subsequent implementation performance of projects that have completed financing, which is the project's actual return. It intends to use empirical research to explore the factors that can affect the returns on ECF projects' investment. The project's financial return can better reflect the quality of the project. ECF backers are most concerned about the project's return. Research on the influencing factors of project returns can contribute to the platform, backers, or fundraisers. This paper aims to fill the current research on ECF's financial profitability gap.

This paper objective is twofold: firstly it expects to improve the current basic theoretical framework of crowdfunding research. Secondly, this research uses traditional linear regression and DNN models to conduct exploratory empirical analysis, focusing on the factors that affect the return on investment of ECF projects. Neural networks have shown clear advantages in some evaluation projects, demonstrating their potential in predicting crowdfunding project funding. This article combines neural networks and Internet finance to provide many practical implications for future research.

## 2. Literature Review

This study analyzes all research on crowdfunding based on data from the Web of Science. According to a review of the existing literature, there are two main research lines on crowdfunding. First, some papers are mainly related to the research of crowdfunding development, such as the definition of crowdfunding, the discussion of the crowdfunding model, and the relationship between crowdfunding and innovative companies and investment [11, 12]. Second, researchers have studied crowdfunding activities' performance and success factors [13, 14]. As for the research on the application of artificial intelligence in crowdfunding, this paper also sorts out the existing research.

The article "Is Equity Crowdfunding the Leapfrog to Companies' Success? Financial Performance in China" was published in 2022. Journal: Comput Intell Neurosci.

### 2.1. Crowdfunding Development and Motivation

Some early studies discussed crowdfunding's definition regarding the first primary research line on crowdfunding development. Belleflamme et al. [1] considered that crowdfunding could be an activity that rewards the backers with experience, services, or products in exchange for financial resources. Based on the previous research, Mollick [11] defined crowdfunding more strictly as a business model where each backer provides a small amount of money and obtains physical goods, services, or equity.

For this main research line, some studies have also focused on the crowdfunding model. They believed that crowdfunding could be divided into four categories: donation-based, reward-based, equity, and lending. Donation-based crowdfunding means backers donate to a project but do not get paid for their support. Reward-based crowdfunding means that project backers can receive nonmonetary rewards for supporting the project. Equity crowdfunding refers to project backers obtaining shares or similar rights of project sponsors by supporting crowdfunding projects. Lending crowdfunding means that project sponsors obtain lower capital costs, and lenders will also have high-return investment opportunities [7, 15]. This classification is also the mainstream view that most scholars now recognize.

Some scholars have focused on the motivations of crowdfunding participants, including backers and project sponsors. Some studies have focused on backer motivation. Belleflamme et al. [16] found that 78% of the backers researched wanted to obtain various returns, such as capital, cash, pre-order products, or services through investments. Kuppuswamy and Bayus [12] considered that when backers demonstrated that their investment would make sense for realizing crowdfunding projects, especially when they are close to their deadline. However, investment motivation will be reduced when the project reaches its stated goal. Similarly, Daskalakis and Yue [17] proposed that young men with higher education are more inclined to invest in crowdfunding projects. Some scholars have also paid attention to the impact of gender on crowdfunding investment. Groza et al. [18] found that female backers are more likely to unite and support same-sex entrepreneurs than male backers.

The article "Is Equity Crowdfunding the Leapfrog to Companies' Success? Financial Performance in China" was published in 2022. Journal: Comput Intell Neurosci.

Some studies have focused on the motivations of project sponsors. Belleflamme et al. [16] discovered that the three main reasons of project sponsors choose crowdfunding, which are financing, exposure, and testing products before entering the market. Some authors also discussed the motivations of project sponsors other than obtaining funding. Bretschneider and Leimeister [19] believed that the motivation of project sponsors is to attract more followers. Cowden and Young [5] found that the project sponsor's motivation was not strictly as positive as it was shown. Some speculators copied and imitated others' projects and gave higher returns to absorb investment. The financing motive for these projects is only fraud.

### 2.2. Performance and Success Factors of Crowdfunding's Internal Activities

The second primary research line mainly covers crowdfunding's internal activities' performance and success factors. Compared with the primary research line, this research line contains more empirical research. Nevertheless, the views of scholars have not yet been unified and even have some contradictory conclusions. It makes it necessary to organize and improve relevant research. Pioneers who started this line, such as Ahlers et al. [7], believed that the geographical distance between backers and project sponsors influences backers' investment decisions, especially in the initial stage of the project financing. Guenther et al. [4] also believed that backers are sensitive to geographic factors. They proposed that the crowdfunding platform has eliminated or reduced some of the economic frictions caused by geographical factors through the Internet.

Another pioneering study with significant influence comes from Mollick [11]. The author found that crowdfunding projects' success was the project's quality, updates, misspellings, and the size of the owner's network. Hobbs et al. [20] emphasized that positive forecast information can bring more investment. Vismara [6] found that disclosing information about professional backers can increase the attractiveness of subsequent investments. Bretschneider and Leimeister [19] pointed out that investment preparation and presentation positively impact the project's success. Financing goals, the running time of the event, and the expected delivery of rewards negatively impact the project's success. Kuppuswamy and Bayus [13] proposed that the lower the frequency of project updates and the higher financing goals, the more difficult it will be to achieve project financing goals. Mahmood et al. [21] found that the more complex the Logo, the more unique it will be and positively impact backers. Calic and Shevchenko [22] believed that project information does not only have a positive or negative monotonous effect on financing performance. Signals of autonomy, innovativeness, competitive aggressiveness, and risk-taking have an inverted U-shaped relationship with crowdfunding performance.

The article "Is Equity Crowdfunding the Leapfrog to Companies' Success? Financial Performance in China" was published in 2022. Journal: Comput Intell Neurosci.

Also, some other studies have focused on the social capital ownership of crowdfunding. Bretschneider and Leimeister [19] found that social relations and interaction with crowds will positively impact the project's success. Richter et al. [14] considered that increasing social activities during the project's financing could increase the success rate of projects. Kuppuswamy and Bayus [13] believed that family roles and social influences would positively impact project success. More recently, Hsieh et al. [23] proposed that crowdfunding projects related to social movements have a higher success rate than general projects. Simon et al. [24] found that social closeness and contact frequency did not increase the investment, while the feelings of obligation and the fear of loss did.

### 2.3. Artificial Intelligence and Crowdfunding

Artificial neural networks are an effective prediction technique. Many existing studies have proved that using neural networks can improve the prediction accuracy of traditional models [25]. Using neural network models to study the influencing factors of the financial performance of ECF is the focus of current research. Existing studies such as Thakial and Arora [25] briefly reviewed the development of artificial neural networks at the current stage. Techniques and applications such as multilayer perceptron, T-S fuzzy neural network, support vector machine, radial basis function network, Levenberg–Marquardt algorithm, and backpropagation are also proposed. They also proposed a neural network-based candidate prediction model for predicting projects for various candidates based on certain parameter ratings.

Existing research provides evidence that deep learning can help predict the outcome of crowdfunding projects in advance. Whether project sponsors, project backers, or crowdfunding platforms can benefit from predicting the outcome. Several studies have focused on using artificial intelligence models to predict the success of crowdfunding projects. Lee et al. [26] built a DNN model with textual data from item descriptions as samples. The results show that their neural network model can predict the success of crowdfunding projects well. Cheng et al. [27] have studied how to predict the success of crowdfunding projects based on neural networks, and they believed that image features in project descriptions are the key. Duan et al. [28] investigated whether an entrepreneur's facial trustworthiness affects the success of a crowdfunding project by using machine learning-based face detection technology. They found that the facial trustworthiness of entrepreneurs positively affected the success of crowdfunding projects, and it was particularly significant in female entrepreneurs.

The article "Is Equity Crowdfunding the Leapfrog to Companies' Success? Financial Performance in China" was published in 2022. Journal: Comput Intell Neurosci.

More recently, Wang et al. [29] introduced a deep learning algorithm (multilayer perceptron) and used it to predict crowdfunding performance. They compare deep learning to other commonly used machine learning algorithms. The experimental results show that the prediction accuracy of the deep learning model for crowdfunding fundraising results is 92.3%, which is satisfactory. Shi et al. [30] used machine learning to study the impact of multimedia information in crowdfunding projects. They demonstrated that artificial intelligence could be used to predict the success of crowdfunding projects by training a machine learning model based on audio analytics. Korzynski et al. [31] focused on artificial intelligence in technology-related videos to predict the success of crowdfunding projects. They found that self-presentation and exemplification techniques positively impacted project success, while intimidation was the opposite.

Some studies also focus on AI's impact on crowdfunding performance. Yuan et al. [32] developed a text analysis-based neural network model, Domain-Constrained Latent Dirichlet Allocation (DC-LDA) topic model, to study the topic features of texts in project descriptions, thereby helping entrepreneurs to screen the most crucial text information in the project description and improve the financing performance of the project. Shafqat and Byun [33] focused on fraudulent activities in crowdfunding projects and used a neural network architecture based on language modeling to classify the content of comments in crowdfunding projects, thereby helping backers find safer and more suitable projects. Raab et al. [34] studied the impact of facial expressions on investment motivation using machine learning based on emotion contagion theory. They found that happy and sad facial expressions were positively correlated with investment motivation, but high-intensity facial expressions were negatively correlated with investment motivation expressions. Peng et al. [35] have studied the application of ensemble-based machine learning algorithms in medical crowdfunding, and they believe that the fundraising amount of medical crowdfunding projects can be predicted by machine learning.

### 2.4. Basic Theory of the Neural Networks

Artificial neural networks mimic the neural way the human brain processes information. It can be trained using sample information to have brain-like memory and recognition capabilities [25]. The neural network signal processing needs to satisfy the following formula:

(1) $$\begin{array}{c} \varphi =y\left(\overset{i}{\underset{j=1}{\sum }}N_{j}{ℱ}_{j}-\beta \right.. \end{array}$$

Input *i* signals in the neuron, through the activation function *y*(*i*) of the neuron, and the threshold *β* of signal processing, the final output signal *φ*, and *N*_*j*_ represents the weight of the input point.

The article "Is Equity Crowdfunding the Leapfrog to Companies' Success? Financial Performance in China" was published in 2022. Journal: Comput Intell Neurosci.

A complete neural network is formed by combining several different neurons at a scientific level and sequence [26]. The neural network generally consists of three parts: input layer, hidden layer, and output layer. The specific structure is shown in Figure 1.

The neural network is a typical topological structure. The research field divides the neural network topology into feedforward neural networks and feedback neural networks. The feedforward neural network adopts a unidirectional multilayer structure. Each neuron is only connected to the neurons in the previous layer, and there is no feedback between layers. In the feedback neural network, neurons not only need to receive signals from other neurons but also need to receive their own feedback signals [26]. We suppose that there are two neurons in the output layer, three neurons in the input layer and the hidden layer, and *x* is the sample size, which is expressed as follows:

(2) $$\begin{array}{c} \text{Train}=\left\{\left(K_{1},M_{1}\right),\left(K_{2},M_{2}\right),\ldots ,\left(K_{x},M_{x}\right)\right\}. \end{array}$$

In the case where each side in the neural network has a weight, we suppose the weight matrix between the hidden layer and the input layer is as follows:

(3) $$\begin{array}{c} Q^{\left[1\right]}=\left[\begin{array}{ccc} a11 & a21 & a31\\ a12 & a22 & a32\\ a13 & a23 & a33 \end{array}\right]. \end{array}$$

The number of rows in the matrix is equal to the number of neurons in the hidden layer, and the number of columns in the matrix is equal to the number of neurons in the input layer.

(4) $$\begin{array}{c} Q^{\left[2\right]}=\left[\begin{array}{cccc} a11 & a21 & a31 & a41\\ a12 & a22 & a32 & a42 \end{array}\right]. \end{array}$$

In the above matrix, the number of rows of the matrix is equal to the number of neurons in the output layer, and the number of columns of the matrix is equal to the number of neurons in the hidden layer. The biases of the hidden layer and the output layer are, respectively, recorded as follows:

(5) $$\begin{array}{c} p^{\left[1\right]}=\left[p1^{\left[1\right]},p2^{\left[1\right]},p3^{\left[1\right]},p4^{\left[1\right]}\right]x^{i},\\ p^{\left[2\right]}=\left[p1^{\left[2\right]},p2^{\left[2\right]},p3^{\left[2\right]},p4^{\left[2\right]}\right]x^{i}. \end{array}$$

With the literature analyzed, the following research question is defined:

RQ1: What factors will affect the return on investment of equity crowdfunding projects in China?

The article "Is Equity Crowdfunding the Leapfrog to Companies' Success? Financial Performance in China" was published in 2022. Journal: Comput Intell Neurosci.

## 3. Context, Variable, and Methodology

### 3.1. Context

This paper uses the project on China's first and the largest ECF platform, “Renrentou” as a sample. In “Renrentou,” all projects must have physical store chains with more than two stores, and the minimum investment of the project part is 10% of its equity. The platform backers are mainly based on ordinary people. Moreover, as one of China's largest civil crowdfunding platforms, it is the only platform that allows us to obtain data on the projects' dividends. Therefore, this paper collected data on 600 projects that have been funded on this platform. Since these data are independent and decentralized, various types of information need to be searched separately and cannot be obtained with tools, so they need to be collected manually.

This paper collected and used quarterly reports instead of annual reports of the projects published on the platform “Renrentou.” Then, this paper found that two companies in the sample have gone bankrupt when collecting sample data. However, their performance has been announced and does not affect this paper.

### 3.2. Variable

Regarding the selection of variables, this paper divides them into three types of influencing factors based on the data collected: the project sponsor company information, the company representative information, and the project-self information.

The project sponsor company's information includes the company's operating time, the number of employees, and the number of branches already opened [11, 13, 21]. The company's operating time (*D*) refers to the years from establishing the project sponsor company to the project's collection deadline (2020). Employees (*E*) refer to the number of existing employees of the project sponsor company. Since the number of employees in a company is continuously changing, the company usually announces its number as an interval value. Therefore, this paper uses the average of the numbers. The number of stores (NT) refers to the number of branches opened by the project sponsor company. This paper only takes the number of its direct stores. Chain stores do not consider it because their assets do not belong to the project sponsor company. These variables are common financial indicators that can reflect the strength of the project sponsor company.

The article "Is Equity Crowdfunding the Leapfrog to Companies' Success? Financial Performance in China" was published in 2022. Journal: Comput Intell Neurosci.

The company representative's information refers to its knowledge level (ES) and gender (SP) collected in this paper. The company representative is the core of the company team. For startups, it often plays a decisive role [17, 18, 20].

For the project-self information, since this study is aimed at ECF projects, the benefits will be more concerned. Therefore, this paper uses the expected rate of return (TRE) announced by the project as a variable, reflecting the project sponsor company's prediction of the project quality. This paper also focuses on the initial investment amount (CII) and financing goal (OC). The initial investment amount refers to the minimum investment amount of the project. The financing goal refers to the expected value of the project sponsor company to raise funds. These two indicators also reflect the quality of the project.

In addition, based on the projects' collected financial data, this paper calculates the actual rate of return, which is the indicator's ROE, which refers to the actual rate of return for project backers. Simultaneously, RCR is calculated based on the currently collected projects' registered capital and total dividends. This paper uses ROE and RCR as profitability indicators because they reflect the true quality of the project. Considering the general situation of the project, their industries have not been distinguished. The ROE calculation method this paper used was the method commonly used in accounting calculated as the net income of a company divided by the total equity of the company. In the data published in these projects, this paper collected their net income and total investment through their quarterly reports to calculate the ROE. However, as these reports often lack many items, it is difficult to calculate other indicators.

### 3.3. Methodology

This paper studies what factors can affect the return of investment on ECF projects in China. Therefore, this paper will use the project's profitability indicators, TRE, and RCR as independent variables. The project announces TRE, reflecting the project sponsor company's expectations of its returns. This paper calculates RCR. It is the total dividend divided by the registered capital to calculate RCR. It is not the same as the ROA used in traditional accounting. Because the registered capital is not the current actual capital, it can also reflect its profitability expectations. Moreover, this study adopts the real rate of return (TRR)/(ROE in accounting) as the dependent variable. As the most direct measurement indicator, it can reflect the real return on investment of the enterprise.

In this paper, the multiple linear regression model is used for testing after using the Poisson model to eliminate the autocorrelation factors between independent variables. This test can reflect whether the two profitability indicators of TRE and RCR can affect the true rate of return, as shown in the following formula:

(6) $$\begin{array}{c} TRR=\beta_{0}+\beta_{1}TRE+\beta_{2}RCR+\varepsilon . \end{array}$$

This paper has found through pretesting that the binary logistic regression model could better explain the *RQ* of this study. Therefore, this paper defines a new independent variable *R*. The independent variable *R* represents the result. When the value of TRR is greater than or equal to TRE's value, *R* is “1,” which means the project is a “success.” When the value of TRR is less than TRE's value, *R* is “0,” indicating that the project failed. Therefore, the research model currently is as follows:

(7) $$\begin{array}{c} R=\beta_{0}+\beta_{1}D+\beta_{2}E+\beta_{3}RCR+\beta_{4}NT+\beta_{5}ES\_\text{yes}+\beta_{6}SP\_\text{woman}+\beta_{7}OC+\beta_{8}CII+\beta_{9}TRE+\varepsilon . \end{array}$$

where *D* is “the company's operating time”; *E* is “number of employees”; *NT* is “the number of branches already opened”; and *ES* is “the knowledge level of company representative, that is, whether the company representative has received higher education.” As a dummy variable, it is divided into “ES_yes” and “ES_no”; *SP* is “gender of company representative,” and as a dummy variable, it is divided into “SP_woman” and “SP_man”; *OC* is “financing goal”; *TRE* is “expected rate of return”; and *CII* is “the initial investment amount.”

The article "Is Equity Crowdfunding the Leapfrog to Companies' Success? Financial Performance in China" was published in 2022. Journal: Comput Intell Neurosci.

In this study, the sample data were preprocessed, and the natural logarithm of all numerical variables was taken to eliminate the effect of scale between variables.

### 3.4. Applicability of the DNN Model

The DNN model is relatively cumbersome and complex, involving a large number of training parameters. How to choose the training method and to obtain the required learning parameters is a key link worthy of in-depth thinking. In the era of artificial neural networks, the depth of the model is at most three layers, and the learning parameters involved are relatively small. It can obtain a completer and more reasonable model through a simple BP algorithm. With this advantage, the BP algorithm is favored and respected by people in the industry, and it has been vigorously promoted and actively applied in many fields. However, BP neural network is not perfect. It also has its limitations. In practical analysis, due to the use of a large number of parameters, the algorithm's search space is huge, resulting in more complex error surfaces, and it is easy to obtain poor local optimal solutions. The experimental sample data are directly related to the final performance of the algorithm. If the sample is poorly representative or contradictory, it is difficult for the model to achieve the expected performance. In training through the BP algorithm, the gradient dispersion phenomenon tends to be further aggravated, affecting the model's performance. Moreover, compared with other neural networks, the operation speed of the BP neural network is slower. For the above problems and deficiencies, pretraining methods can be used to avoid them. Exploiting unlabeled data in an unsupervised form provides objective and accurate initial parameters for subsequent training. Satisfactory results can be obtained even with very little labeled data. Given the problems of the recurrent neural network, the farther the node is from the current node, the effect of the current node processing gets smaller and smaller. However, this paper considers that the data parameter dimension in this paper is not constrained in terms of efficiency. Therefore, the DNN model established in this paper corresponds to the formula (7) in this paper, and the output layer is the binary logic result, that is, the “success” or “failure” of the crowdfunding project.

The article "Is Equity Crowdfunding the Leapfrog to Companies' Success? Financial Performance in China" was published in 2022. Journal: Comput Intell Neurosci.

## 4. Results

### 4.1. Traditional Linear Regression Analysis

The first test tests the impact of the two profitability indicators selected in this paper on the project's profitability expectations. We have used model (6) to perform the regression; the results are shown in Table 1.

First, the *R*-square value is 0.180, and the (6) adjusted *R*-square value is 0.171. Since the equation in this paper belongs to the explanatory regression equation in social sciences, 17.1% descriptive degree has specific statistical significance (similarly, [11] proposed the optimal R-square among the six models in his research is 0.18). Durbin–Watson's value is 1.772, which indicates that the variables in this article have no serial correlation, and the equation is not a pseudoregression. Since the Sig. values of LnRCR and LnTRE are 0.000 and 0.013, both are less than 0.05. We reject the null hypothesis within the confidence interval of *P* = 0.05. That is, both independent variables can significantly affect the dependent variable TRR.

The coefficient B value of the independent variable return on registered capital (LnRCR) was 0.207, indicating a significant positive correlation with the dependent variable actual rate of return (TRR). This shows that the higher the RCR of the project sponsor company, the higher the actual rate of return. This is consistent with the speculation in this paper when selecting variables. The higher the expected value of the project's profitability, the more the actual returns. The B value of LnTRE is −0.231, hurting RTS the dependent variable TRR. This means that the higher the expected rate of return of the project sponsor company, the lower the project's actual return. This result also reflects that project sponsors may overestimate their projects' quality and set excessive project return expectations to attract backers. Moreover, this negative effect shows that this phenomenon is not an exception in this paper's samples.

The article "Is Equity Crowdfunding the Leapfrog to Companies' Success? Financial Performance in China" was published in 2022. Journal: Comput Intell Neurosci.

The second test in this paper tests the effect of all independent variables on return on investment. In this part, this paper uses the binary logistic regression model that is the model (7) for analysis.

According to the definition of this research, the R-value is 1 equal to the project “success,” and the *R*-value is 0 means the project “failure.” As shown in Table 2, “success” occurred 90 times, and “failure” appeared 510 times. The research model of this paper simulates the overall prediction accuracy of 90.0%.

Table 3 reflects the degree of influence of independent variables on dependent variables. The value of the *R*-squared of Cox and Snell is 0.260, indicating that the degree of interpretation of the independent variable by the dependent variable is 26.0%. Nagelkerke's *R*-square value is 0.455, which shows that the model in this paper is meaningful.

The results in Table 3 show that the project sponsor company's operating time has a statistically significant positive effect on the investment return within the confidence interval of *P* value of 0.05. This implies that the longer the project sponsor's company has been operating, the more likely the actual rate of return of the project will reach the expected rate of return. This result confirms the suspicion of variable selection in this paper that companies with power can only operate for a long time. By contrast, companies lacking power cannot operate sustainably.

Surprisingly, the results found that the number of employees of the project sponsor company and the return on investment was statistically negatively correlated within a confidence interval of a *P* value of 0.05–0.10. The number of employees of the project sponsor company has a statistically negative effect on the investment return within the confidence interval of *P* value of 0.05–0.10. This means that the greater the number of employees in the project sponsor company, the more difficult it is for the actual rate of return of the project to reach the expected rate of return. This result is contrary to the speculation of variable selection in this paper. Although not a statistically significant negative correlation, this result is also noteworthy. This paper speculates on the reason for this result, which may be due to a large number of employees, making the company's management more difficult. However, this paper cannot determine the specific cause of this phenomenon.

The article "Is Equity Crowdfunding the Leapfrog to Companies' Success? Financial Performance in China" was published in 2022. Journal: Comput Intell Neurosci.

The knowledge level of the company representative has a statistically negative effect on the investment return within the confidence interval of *P* value of 0.05–0.10. This implies that if the company representative of the project sponsor company has received higher education, their project's actual rate of return is more challenging to achieve the expected rate of return. This result is inconsistent with common sense. This paper speculates that this phenomenon may be because the highly educated company representative overestimated the project's rate of return.

The expected rate of return of the project has a statistically significant negative effect on the investment return within the confidence interval of a *P* value of 0.05. That shows that the higher the expected rate of return of the project, the more difficult it is to achieve the actual rate of return of the project. This result also reflects that the project sponsor may overestimate the quality of its project, making it difficult for the actual rate of return to reach the expected rate of return they have announced. The research of Cowden and Young [5] also had similar results. They found that some speculators' projects only care about the amount of financing, not the project's quality. These projects give backers false and generous return signals, but these projects did not perform well after financing.

The registered capital return has a statistically positive effect on investment return within the confidence interval of *P* value of 0.05–0.10. When the project's registered return on capital is higher, the project's expected rate of return is more likely to be reached. This result also confirms the speculation in the selection of variables in this paper. This profitability indicator reflects the real quality of the project. A company with higher profitability is more likely to succeed in the project.

### 4.2. Deep Neural Network Analysis

The establishment of the DNN model structure in the research is built using the Keras framework. Keras is a deep learning API written in *Python*, and it can speed up the training of the model [36]. In this model, the selected neuron activation function is the ReLU function. The ReLU function is the most used activation function in deep learning model training, it is relatively simple to calculate, and it is easier to optimize when the operation of the neural network model is linear or close to linear. The loss function in this study is cross-entropy, Adam is chosen by the iterative optimizer, and the connection weights and biases of each layer are initially randomly generated. For the training of the model, after synthesizing the literature and the actual situation, this paper decides that the number of times each training is 50, with a total of 10 iterations, and the model is evaluated after the training. This paper considers the model by outputting the loss function value of the DNN model and the accuracy of the test set.

The article "Is Equity Crowdfunding the Leapfrog to Companies' Success? Financial Performance in China" was published in 2022. Journal: Comput Intell Neurosci.

As shown in Figure 2, the experimental results of the DNN model shown in the above figure show that after only 10 times of training, the accuracy rate on the test set has reached 86.4%. This good prediction effect preliminarily proves that the DNN model can be applied in the research field of success factors of Internet ECF projects. Therefore, in the following work of this paper, the number of training will be increased to observe the prediction accuracy after training.

This research uses the Python deep learning framework as a tool to build DNN-based success factors for the ECF identification model. In this paper, the data are made according to the ratio of the training set and the test set to 2 : 1. After the production, there are 400 training sets and 200 test sets. To maintain consistency with the regression experiments in 4.1 of this paper, this paper defined two types of ECF projects: “failures” or “success.” So, the class of the output layer is 2, and a SoftMax classifier is used to calculate the output probability for each category. The schematic diagram of the ReLU activation function expression used is shown in Figure 3, and the expression is as follows:

(8) $$\begin{array}{c} y\left(u\right)=\frac{1}{1+c^{u}}. \end{array}$$

Then, we set the hyperparameters, the learning rate is set to 0.001, the number of iterations is set to 40, the number of batches for each processing is 10, and the loss function selects the cross-entropy loss function, and the training method is retraining. During the training process, we always need to pay attention to the changes in the two parameters of loss and accuracy. The loss curve and accuracy curve of the built DNN model are shown in Figure 4.

As seen from the loss graph shown in Figure 4(a), there are two curves in the figure, and the change trends of the two curves are basically the same. It starts to drop rapidly from the loss value of about 1, and after 25 iterations, the curve declines slowly. Then, the curve gradually becomes stable after 100 times. It shows that the network begins to converge, the training is completed after 200 rounds, and the loss value drops below 0.6.

The article "Is Equity Crowdfunding the Leapfrog to Companies' Success? Financial Performance in China" was published in 2022. Journal: Comput Intell Neurosci.

From the accuracy curve shown in Figure 4(b), the training accuracy curve of the DNN network increases significantly with the increase of the number of iterations. It starts to slow down around 15 rounds, and as the level increases, it converges at around 80 rounds, and the accuracy rate reaches 100%, and it remains stable until the end of the training. The changing trend of the test accuracy rate is slightly different. The accuracy rate starts to rebound sharply at 60% in the 5th round and is roughly the same as the changing trend of the training accuracy rate, reaching 95% in the 14th round. After the hierarchical increase, it converged in about 60 rounds, and the accuracy rate went to 98.5%, and it remained stable until the end of the training. It can be seen from the loss curve and accuracy curve that the DNN network converges stably. As can be seen from the accuracy and loss values, the generated model performs better.

After it is concluded that the generated model is convergent and has good performance, the verification analysis of the developed classification model is carried out, and some common indicators test the model performance. The first is the confusion matrix analysis. From the production of the data set, there are 200 data in the test set. The classification results of the data are shown in Table 4.

After the model operation, the prediction results can be seen in Table 4. Through this table, we can clearly and intuitively understand that the total error of DNN classification is about 3%, which clearly shows that DNN has a decisive advantage in predicting ECF projects. Compared with the 90% accuracy of the prediction results of the logistic regression model in this paper (shown in Table 2), the DNN model in this paper predicts 97% better performance.

ROC (receiver operating characteristic curve) is a comprehensive index reflecting continuous variables of sensitivity and specificity, and each point on it reflects the sensitivity to the same signal stimulus. In this study, the ROC curve can reflect the binary classification prediction results of the neural network model. Generally, the image plane area between the ROC curve and the coordinate axis is used as an important indicator to evaluate the prediction accuracy of the model, and the higher the value, the better the prediction accuracy.

AUC (area under curve) is defined as the size of the area enclosed by the coordinate axis under the ROC curve, and the value ranges from 0.5 to 1. The closer the value of AUC is to 1, the higher the real degree of its use method, and when the AUC is equal to 0.5, it means that it has no practical value. In Figure 5, the AUC values of category 0 and category 1 are 0.995 and 0.992, respectively, and close to 1. When the AUC value is closer to 1, the model performs better. It can be seen that the performance of the DNN model proposed in this paper is relatively good.

The article "Is Equity Crowdfunding the Leapfrog to Companies' Success? Financial Performance in China" was published in 2022. Journal: Comput Intell Neurosci.

This research uses the ROC package in the *R* language to draw random forests, decision trees, and support vector machine of ROC curves, as shown in Figure 6.

As shown in Figures 6(a)–6(c), after calculation, the predicted AUC values of random forest three classifications are 0.99 and 0.97. The three-category prediction AUC values of the decision tree were 0.98 and 0.89. The support vector machine's three-category prediction AUC values were 0.996 and 0.98. Compared with the above results, the three-category prediction AUC value of the DNN algorithm has the best effect and the highest accuracy. In particular, category 1 is significantly higher than other algorithms. It shows that the DNN model has exceptionally high sensitivity and accuracy in identifying ECF project success.

At the same time, to minimize the impact of the different distribution of training samples on the accuracy of model analysis, this research uses the tenfold cross-check method to test the model's fur. First, we divided the research index data into ten parts on average, then defined nine index data as datasets according to a particular order. The selected data were used for testing, and ten repeated results were obtained. The average misjudgment rate was used to measure the pros and cons of the DNN for ECF projects.

It can be seen from Figure 7, and the average model prediction accuracy of category 0 and category 1 is all around 95%. It can be seen that the prediction accuracy of the model is high, which shows the validity and objectivity of the sample classification.

According to Table 5, factors such as the company's operating time, number of employees, expected rate of return, and the actual rate of return that can be borne have an important impact on the success of the ECF project. Among them, the company's operating time and the expected rate of return have the most significant effect on ECF projects. The results are similar to our results in the linear model (7).

## 5. Conclusions

Crowdfunding is an thrilling and innovative field. In recent years, more and more scholars have begun to pay attention to ECF. Through the review of existing research, this paper found that crowdfunding research is divided into two main research lines. One is related to the development of crowdfunding. It includes the definition of crowdfunding, the classification of crowdfunding platform models, and the motivations of crowdfunding participants. The other is the research on the performance and success factors of crowdfunding's internal activities, mainly about the project's success factors and the research on various kinds of crowdfunding information. In addition, the application of artificial intelligence in crowdfunding has had a strong development potential.

The article "Is Equity Crowdfunding the Leapfrog to Companies' Success? Financial Performance in China" was published in 2022. Journal: Comput Intell Neurosci.

In the empirical research part, this paper found that the expected rate of return and the return on registered capita indicators defined by this paper can significantly impact the actual rate of return. It proved that the profitability index calculated using financial data could reflect the project's real quality. However, the negative impact of the expected rate of return, this paper considers that project sponsors may overestimate project quality and set high project return expectations to attract investors.

For the logistic regression model, the results show that companies which can operate for a long time are more powerful, and companies with certain strengths are more able to formulate a reasonable and achievable expected rate of return. Thus, it is easier to achieve success. In addition, the paper finds that an excessive number of employees can make the company's management more difficult. This will affect the healthy operations of the company and lead to poor financial conditions that make it difficult to achieve success. Also, this paper found that highly educated company representatives could overestimate the rate of return of the project. Moreover, this paper estimates that company representative with no higher education is more willing to show backers the project's actual situation, and their entrepreneurial goals appear more authentic.

Besides, this paper proposes to use a DNN model to gradually identify and predict the influencing factors that affect the success of the financing. It also trains and indicates the model to obtain better training prediction results. It proves that the prediction performance of the DNN model on the ECF factor of success is relatively good. After the verification and analysis of the classification evaluation index of the DNN model, it shows the scientific, objectivity, and rigor of the empirical evidence, using cross-validation with other classification models. It shows that compared with the traditional regression model, random forest, support vector machine, and decision tree, the comprehensive effect of the DNN model is the best, and the accuracy is the highest.

This article does not discuss the reasons for such a low success rate. However, Cowden and Young [5] pointed out one of the shocking reasons in their research: some entrepreneurs steal others' ideas to absorb investment and use ECF to deceive backers. For ECF, although there is still no way to eliminate these “junk” projects, the transparency of projects increases as the industry develops and matures. The industry's supervision improves, and the quality of the projects will also improve.

The article "Is Equity Crowdfunding the Leapfrog to Companies' Success? Financial Performance in China" was published in 2022. Journal: Comput Intell Neurosci.

However, this paper cannot trace and characterize the specific impact reasons for all the results. It is also one of the research limitations of this article. Another limitation is that the ECF project has not been able to obtain the complete financial statements of the project. This paper is based on a few original financial variables. The research on ECF projects' financial transparency will become one of the new goals of ECF research in the future. More transparent financial statements can encourage backers to invest, but from a macroperspective, they can also contribute to the sustainable development of the crowdfunding industry.

## Figures and Tables

**Figure 1:** Schematic diagram of neural network structure.

**Figure 2:** Prediction results of DNN after 10 times of training.

**Figure 3:** ReLU function diagram.

**Figure 4:** The loss curve and accuracy curve of the neural network model.

**Figure 5:** ROC curve and AUC value.

**Figure 6:** ROC curve and AUC value.

**Figure 7:** Tenfold cross-check results.

**Table 1:** Regression results for model.

Model (7)	Unstandardized coefficients		Standardized coefficients	*t*	Sig.	*R* square	Adjusted *R* square	Durbin–Watson
	B	Std. Error	Beta					
Constant	−2.316	0.176		−13.148	0.000	a		
LINT (LnRCR)	0.207	0.033	0.409	6.271	0.000	0.180	0.171	1.772
LINT (LnTRE)	−0.231	0.092	−0.164	−2.517	0.013			

**Table 2:** Classification table.

Classification table					
Observed		Predicted		
		Result		Percentage correct
		Failure	Success	
Step 1	Result	Failure	495	15	97.0
		Success	45	45	50.0
	Overall percentage				90.0
a. The cutoff value is 0.500					

**Table 3:** Regression results for model.

Model (8)	*B*	S.E.	Wald	d*f*	Sig.
LnD	**1,384**	,549	6,354	1	**,012**
LnE	−**,492**	,297	2,743	1	**,098**
LnNT	−,011	,163	,004	1	,947
ES_YES	−**,940**	,533	3,106	1	**,078**
SP_WOMAN	−,693	,798	,754	1	,385
LnOC	−,172	,329	,274	1	,601
LnCII	,260	,498	,273	1	,601
LnTRE	−**1,526**	,285	28,571	1	**,000**
LnRCR	**,190**	,108	3.088	1	**,079**
Constant	−2,651	4,315	,377	1	,539
−2 log likelihood	108.763^a^				
Cox and Snell *R* square	0.260				
Nagelkerke *R* square	0.455				

**Table 4:** Neural network model confusion matrix.

		Forecast result		
		0	1	Percentage
The actual situation	0 (failures)	167	13	98.2
	1 (success)	27	3	90.0
	Overall percentage			97.0

**Table 5:** Importance of features.

Feature	Importance
*D*	13
*E*	−5.8
RCR	3
NT	−1.6
ES	−6
SP	−0.6
OC	−0.1
CII	0.1
TRE	−14

The article "Is Equity Crowdfunding the Leapfrog to Companies' Success? Financial Performance in China" was published in 2022. Journal: Comput Intell Neurosci.

## Data Availability

The data that support the findings of this study are available from the corresponding author upon reasonable request.
